# Co-Expression of Foreign Proteins Tethered to HIV-1 Envelope Glycoprotein on the Cell Surface by Introducing an Intervening Second Membrane-Spanning Domain

**DOI:** 10.1371/journal.pone.0096790

**Published:** 2014-05-07

**Authors:** Hongyun Wang, Xiao Li, Shuhei Nakane, Shujun Liu, Hirohito Ishikawa, Aikichi Iwamoto, Zene Matsuda

**Affiliations:** 1 China-Japan Joint Laboratory of Structural Virology and Immunology, Institute of Biophysics, Chinese Academy of Sciences, Beijing, China; 2 University of Chinese Academy of Sciences, Beijing, China; 3 Research Center for Asian Infectious Diseases, Institute of Medical Science, the University of Tokyo, Tokyo, Japan; 4 Division of Infectious Diseases, Advanced Clinical Research Center, Institute of Medical Science, the University of Tokyo, Tokyo, Japan; Institute of Infection and Global Health, United Kingdom

## Abstract

The envelope glycoprotein (Env) of human immunodeficiency virus type I (HIV-1) mediates membrane fusion. To analyze the mechanism of HIV-1 Env-mediated membrane fusion, it is desirable to determine the expression level of Env on the cell surface. However, the quantification of Env by immunological staining is often hampered by the diversity of HIV-1 Env and limited availability of universal antibodies that recognize different Envs with equal efficiency. To overcome this problem, here we linked a tag protein called HaloTag at the C-terminus of HIV-1 Env. To relocate HaloTag to the cell surface, we introduced a second membrane-spanning domain (MSD) between Env and HaloTag. The MSD of transmembrane protease serine 11D, a type II transmembrane protein, successfully relocated HaloTag to the cell surface. The surface level of Env can be estimated indirectly by staining HaloTag with a specific membrane-impermeable fluorescent ligand. This tagging did not compromise the fusogenicity of Env drastically. Furthermore, fusogenicity of Env was preserved even after the labeling with the ligands. We have also found that an additional foreign peptide or protein such as C34 or neutralizing single-chain variable fragment (scFv) can be linked to the C-terminus of the HaloTag protein. Using these constructs, we were able to determine the required length of C34 and critical residues of neutralizing scFv for blocking membrane fusion, respectively.

## Introduction

HIV-1 envelope glycoprotein (Env) mediates membrane fusion between the viral and cell membranes. Env is first synthesized as gp160 precursor protein, and then cleaved into gp120 and gp41 in Golgi apparatus. After cleavage, gp120 and gp41 remain non-covalently associated and form trimetric spikes [1], [2], [3]. The gp41 subunit is a transmembrane protein composed of an ectodomain, a single membrane-spanning domain (MSD) and a cytoplasmic domain [4], [5], [6]. Binding of gp120 to the CD4 receptor and co-receptor (CXCR4 or CCR5) triggers the conformational changes of gp41, which mediate membrane fusion process [7], [8], [9]. HIV-1 Env has been a major target of anti-viral strategies such as the development of fusion inhibitors and anti-HIV vaccines [10], [11], [12], [13], [14].

To achieve a quantitative cell-cell membrane fusion assay, we recently developed a new pair of reporter proteins called dual split proteins (DSPs) [15], [16]. We have used DSP assay to determine the co-receptor usage of the HIV-1 isolates [17]. DSP assay can be applied to the analysis of the mutants of envelope proteins of HIV-1 Env [15], [18] or other virus [19]. For such an assay, it is desirable to determine the level of HIV-1 Env expressed on the cell surface [20], [21], [22]. The commonly used method is an immunological staining of HIV-1 Env with a specific antibody. However, the limited availability of universal antibodies that can recognize naturally divergent HIV-1 Envs as well as laboratory-made mutant Envs is a problem. To overcome this technical difficulty, here we explore the possibility to link a tag protein called HaloTag to HIV-1 Env. HaloTag is a newly developed tag that can be covalently labeled with either a membrane-permeable or impermeable ligand conjugated with a fluorescent chromophore [23]. We have previously utilized HaloTag to examine the membrane topology of gp41 [24]. In this study, to use HaloTag as a surrogate surface marker, we introduced an MSD derived from human transmembrane protease serine 11D (TM11D) between the C-terminus of gp41 and the N-terminus of HaloTag.

The introduction of the second MSD successfully relocated the connected HaloTag to the cell surface and did not compromise the fusogenicity of Env drastically. By probing HaloTag with a membrane-impermeable fluorescent ligand, the level of Env expressed on the cell surface can be estimated indirectly. Using this surface level of Env, the fusion activity can be normalized. We showed that an additional peptide or protein such as scFv was able to be connected to the C-terminus of the HaloTag. This allowed us to characterize the critical residues of neutralizing scFvs.

## Results

### The Second Membrane-spanning Domain between the C-terminus of gp41 and Following HaloTag Relocates the HaloTag onto the Cell Surface

We introduced a 21 aa-long MSD derived from transmembrane protease serine 11D (TM11D; *Homo sapiens*), a type II membrane protein, as a second MSD (MSD2) after the gp41 cytoplasmic tail. Attaching the MSD of TM11D and HaloTag to the C-terminus of Env produced the HXB2-TM11D-Halo construct (Fig. 1A). The *env* gene of HXB2 origin used in this study was codon-optimized for mammalian expression. To test whether introduction of the MSD2 successfully flipped out the tethered HaloTag protein, staining of HaloTag with specific ligands with different membrane permeability was applied. The membrane-permeable TMR ligand can penetrate membranes and label all HaloTag both in and out of the cells, whereas membrane-impermeable Alexa Fluor 488 (AF488) ligand only labels HaloTag expressed on the cell surface. Positive AF488 staining was observed for constructs containing TM11D MSD (Fig. 1B). In contrast, the construct without TM11D MSD (HXB2-Halo) was not labeled with AF488, while the intracellular Env-Halo protein was clearly labeled with the membrane-permeable TMR ligand (Fig. 1B). These results clearly showed that the MSD of TM11D linked to the C-terminus of Env was able to translocate downstream HaloTag into the extracellular compartment. In DSP assay, the fusogenicity of HIV-1 Env tagged with HaloTag via TM11D was retained, even after labeling with HaloTag TMR or AF488 ligands, this fusogenicity was not altered (Fig. 1C).

**Figure 1:** Connection of HaloTag to Env with the addition of the intervening second MSD. (A) Upper panel: Design of the Env-TM11D-Halo construct. A CMV promoter drives the expression of the tethered construct in all expression vectors. The 21 aa MSD of TM11D was added to the C terminal of gp41 as an MSD2 to help flipping out the HaloTag. Lower panel: Design of the Env-Halo construct, the control tethered construct without the MSD2 of TM11D. The expected membrane topology of the expressed protein with each construct is depicted schematically on the right. ED: ectodomain of gp41, MSD: membrane-spanning domain of gp41, CT: cytoplasmic tail of gp41. The sequences for Env corresponding to HXB2 or JRFL were used. (B) Confocal microscope analysis of tethered HaloTag in transfected 293FT cells stained with membrane-permeable (TMR, red color) or impermeable (AF488, green color) ligands. The transfected DNA is indicated: Mock, control DNA transfection; HXB2-Halo, Halo directly connects with gp41 (without the MSD of TM11D); HXB2-TM11D-Halo, a construct with the MSD of TM11D added between Env and Halo. Scale bar = 20 µm. (C) Effect of Halo ligands on the fusogenicity of HaloTag attached Env by DSP assay. Halo TMR and AF488 ligands were used to label the HXB2-TM11D-Halo fusion protein. The effect on the fusion activity was measured by DSP assay, which measures pore formation during cell-cell fusion by split *Renilla luciferase* (RL) reporter proteins. DSP activities for the ligand-labeled Env were compared with the HXB2-TM11D-Halo and non-tethered HXB2 Env protein without labeling (only add DMEM culture medium, and the value of HXB2-TM11D-Halo was set at 100%). Error bars represent standard deviations of the results of triplicate experiments. Student’s *t*-test was used to determine the statistical significance of the measured variables for each differently labeled (open column) and the non-labeled (solid column). ns = nonsignificant.

### Staining the Linked HaloTag with the Membrane-impermeable Ligand can be used to Determine the Surface Expression Level of Env

To show the usefulness of the linked HaloTag for estimation of the surface expression level of Env, we performed flow cytometry analysis using the transfected cells. We constructed an expression vector, JRFL-TM11D-Halo similar to HXB2-TM11D-Halo by replacing the *env* gene of HXB2 with that of JRFL, a CCR5-tropic HIV-1. We compared the efficiency of labeling between HaloTag ligand and an anti-HIV-1 V3 antibody.

We transfected 293FT cells with HXB2 Env tethered with HaloTag (HXB2-TM11D-Halo), untethered HXB2 Env (HXB2-WT), tethered JRFL Env (JRFL-TM11D-Halo), untethered JRFL Env (JRFL-WT) or Mock DNA. The surface level of Env was estimated by indirect staining of HaloTag or direct immunological staining of Env. For HaloTag staining, live cell staining with the membrane-impermeable HaloTag AF488 ligand was used for surface labeling and membrane permeable HaloTag Oregon Green ligand was used for the total labeling, respectively. The immunological staining was done with anti-V3 monoclonal antibody V3-G2-25 [25]. Labeled samples were subjected to flow cytometry. Tethered Env stained by membrane-impermeable HaloTag AF488 ligand showed much higher labeling intensity than that of V3-G2-25 antibody labeling (Fig. 2A, 2B). Both surface Env derived from HXB2- and JRFL-constructs were stained well with HaloTag AF488 ligand: about 20% and 40% for HXB2 and JRFL, respectively (Fig. 2D). On the other hand, V3-G2-25 stained HXB2-construct relatively well (12% for HXB2-TM11D-Halo and 27% for HXB2-WT, respectively, Fig. 2D), but the staining of JRFL-construct was very low (both JRFL-TM11D-Halo and JRFL-WT). Halo ligand staining can achieve more general staining than the immunological staining with a specific antibody. In the data shown here, the surface expression level of JRFL Env seems higher than that of HXB2 Env (Fig. 2A). However, it is likely that this is due to higher total expression level of JRFL-construct than that of HXB2-construct, as indicated by the higher staining with membrane-permeable HaloTag ligand (Oregon green) (Fig. 2C, 2D). It seemed that the addition of the second transmembrane domain and HaloTag decreased surface expression level of HXB2 Env, because 27% of cells transfected with untethered HXB2 Env (HXB2-WT) was stained by V3-G2-25, while 12% of cells transfected with tethered HXB2 Env (HXB2-TM11D) was labeled by V3-G2-25 (Figure 2D).

**Figure 2:** Flow cytometry analysis of Env-expressing cells labeled with Halo ligands or anti-Env monoclonal antibody. (A–C) Flow cytometry analysis of Env expression level using different staining strategies. 293FT cells were transfected with expression vectors for tethered Env (HXB2-TM11D-Halo, red line; JRFL-TM11D-Halo, blue line), untethered Env (HXB2-WT, red dashed line; JRFL-WT, blue dashed line), or Mock DNA (grey shade). Cells were stained with membrane-impermeable HaloTag AF488 ligand (A), membrane-permeable HaloTag Oregon Green ligand (C) and anti-Env V3 antibody V3-G2-25 (B). Histograms are representative results from three independent experiments. (D) Positive staining rate of HaloTag labeling and anti-Env antibody immunolabeling of cells transfected with HXB2-TM11D-Halo (solid red bar), HXB2-WT (red shade bar), JRFL-TM11D-Halo (solid blue bar), JRFL-WT (blue shade bar) or Mock (solid gray bar). Error bars represent standard deviations of the results from three independent experiments.

### C34 Peptide Linked to the C-terminus of HaloTag Blocks the Membrane Fusion

Next, we tested whether additional peptide or protein can be linked to the C-terminus of HaloTag to evaluate their biological activities. First, the DNA sequence that encodes C34 was cloned after the HaloTag sequence in the HXB2-TM11D-Halo construct (HXB2-TM11D-C34) (Fig. 3A). C34 is derived from C-terminal heptad-repeat regions (CHR) of gp41 and known to inhibit HIV-1 Env-mediated membrane fusion by interfering with formation of the six-helix bundle [11], [26], [27], [28]. Another peptide 2N derived from the second extracellular loop of chemokine receptor type 5 (CCR5) was introduced as a negative control (HXB2-TM11D-2N), since it has no fusion inhibitory activity [29]. The expression and processing of tethered fusion protein was confirmed by immunoblotting analysis with anti-gp120 and anti-gp41 antibodies (data not shown).

**Figure 3:** Measurement of fusion inhibition of tethered C34 evaluated by syncytia formation and DSP assay. (A) Left panel: Schematic view of HIV-1 gp41. FP, fusion peptide; NHR, N-terminal heptad repeat region; CHR, C-terminal heptad repeat region; MSD, membrane-spanning domain; CT, cytoplasmic tail. The residues are numbered according to their position in HXB2 gp160. The amino acid sequence of C34 is shown. Right panel: The expected membrane topology of HXB2-TM11D-C34 is depicted schematically. (B) Syncytia formation assay in transfected 293CD4 cells. 293CD4 cells were transfected with the indicated constructs (HXB2-TM11D-Halo, HXB2-TM11D-2N, and HXB2-TM11D-C34). After 16 h, the nuclei of cells were stained with Hoechst, and the membrane was stained with CellMask Deep Red plasma membrane stain. White arrows indicate typical syncytia formed in transfected 293CD4 cells. Scale bar = 50 µm. (C) Relative fusion activity was quantified using a fusion index (see Materials and Methods). Fusion activities for each plasmid are shown after normalization to that of the non-tethered Env expression construct (HXB2-WT). The activity of HXB2-WT was set at 100%. Error bars represent standard deviations of the results of five fields. Student’s *t*-test was used to determine the statistical significance of the measured variables for each construct (open column) and control (solid column). Statistical significance was indicated when p<0.001 (***). ns = nonsignificant. (D) Fusion activity measured by DSP assay. Relative fusion activity was measured by DSP assay. DSP activities for each construct were compared with that of the non-tethered Env expression construct (HXB2-WT was set at 100%). Error bars represent standard deviations of the results of triplicate experiments. Student’s *t*-test was used to determine the statistical significance of the measured variables for each construct (open column) and control (solid column). Statistical significance was indicated when p<0.01 (**). ns = nonsignificant.

To examine the effect of the tethered peptides on envelope-mediated cell-cell fusion, a syncytia formation assay was performed in 293CD4 cells. To visualize the generated syncytia clearly, Hoechst 33342 and CellMask Deep Red plasma membrane dye were used to stain the nuclei and plasma membrane, respectively. As expected, cells transfected with the tethered C34 showed no syncytia formation. In contrast, transfection of the HXB2-TM11D-2N construct into 293CD4 cells did not block syncytia formation (Fig. 3B). The level of the syncytia was similar to that of HXB2-TM11D-Halo that does not have any tethered peptide sequence (Fig. 3B). The degree of the syncytia formation was expressed with the fusion index (Fig. 3C). It reflects both the number of syncytia and number of nuclei included in each syncytium [18], [30]. When we used the Env-C34 vector in which the preceding MSD2 sequence was removed (construct with C34 after HaloTag in Env-Halo, see Fig. 1A), the attached C34 failed to prevent syncytia formation (data not shown). These data suggest that the translocated peptide fusion inhibitor was responsible for the observed blockage of syncytia formation.

To further investigate the mechanism of inhibition of membrane fusion by tethered peptide inhibitors, a DSP assay was employed (Fig. 3D). It measures the degree of pore formation and content mixing during cell-cell fusion. Consistent with the syncytia formation assay, HXB2-TM11D-Halo and HXB2-TM11D-2N were positive with DSP assay, while tethered C34 completely inhibited DSP activity (Fig. 3D). This result suggests that C34 blocks pore formation.

### Functional Analysis of Nested Serial C-terminal Deletion Mutants of C34

We examined the effect of truncated CHR-related peptides (C-peptides) on fusion ability by making serial deletion mutants in the HXB2-TM11D-C34 construct. C34 was serially truncated from the C-terminus every two amino acid residues to generate C32, C30, C28, C26 and C24 constructs (Fig. 4C). The ability to block fusion was evaluated by syncytia formation assay and DSP assay (Fig. 4A, 4B). The length of C-peptide correlated well with the ability to block membrane fusion. Tethered C28 began to lose its ability to block membrane fusion, and tethered C24 showed about 30% recovery of membrane fusion compared with HXB2-TM11D-Halo (Fig. 4A, 4B).

**Figure 4:** Measurement of fusion inhibition of nested serial C-terminal deletion mutants of C34 by syncytia formation and DSP assay. (A) Syncytia formation assay in transfected 293CD4 cells. 293CD4 cells were transfected with the indicated constructs (HXB2-TM11D-C24, C26, C28, C30, C32, C34, and HXB2-TM11D-Halo). Relative fusion activity was quantified using a fusion index. Fusion activities for each plasmid are shown after normalization to that of the HXB2-TM11D-Halo construct (set at 100%). Error bars represent standard deviations of the results of five fields. Student’s *t*-test was used to determine the statistical significance of the measured variables for each construct (open column) and control (solid column). Statistical significance was indicated when p<0.001 (***). (B) Fusion activity measured by DSP assay. The relative fusion activity was measured by DSP assay. DSP activities for each construct were compared with that of the HXB2-TM11D-Halo construct (set at 100%). Error bars represent standard deviations of the results of triplicate experiments. Student’s *t*-test was used to determine the statistical significance of the measured variables for each construct (open column) and control (solid column). Statistical significance was indicated when p<0.01 (**) or p<0.001 (***). (C) Amino acid sequence of all C-terminal deletion mutants of C34 are listed.

### Tethered Neutralizing Antibodies can Efficiently Block Syncytia Formation

We replaced the C-peptide with scFv to test whether protein rather than peptide can be introduced after HaloTag. To generate the tethered antibody display constructs, sequences encoding scFvs derived from antibodies b12 (anti-gp120), 2F5 (anti-gp41), and 13H11 (anti-gp41) were cloned to the C-terminal end of HaloTag in the Env-TM11D construct. The b12 antibody binds to the CD4 receptor-binding site of gp120, and 2F5 binds to a linear epitope of membrane-proximal external region (MPER) of gp41 [31], [32], [33], [34]. The antibody 13H11 partially shares its binding site with 2F5 in the gp41 MPER but lacks neutralizing activity, hence served as a negative control [35], [36]. Another small peptide tag (3×FLAG) was placed after scFv for the immunoblotting analysis. Figure 5A shows immunoblotting analysis of the expressed HXB2-TM11D-Halo and HXB2-TM11D-scFv fusion proteins in transfected 293FT cells. The anti-gp120 antibody detected both the precursor gp160 and processed gp120 bands in the wild type Env (Fig. 5A, upper panel, WT). The molecular weight of the precursor form of gp160-TM11D-Halo fusion protein is approximately 200 kDa, and that of gp160-TM11D-scFvs is approximately 230 kDa. Bands with the expected size were observed in each cell lysate, but similar to the WT, the band corresponding to gp120 was weakly detected. To verify processing of the gp160 form into the gp120 and gp41 forms, an anti-FLAG antibody was used. Bands corresponding to the gp160 precursor form (HXB2-TM11D-scFvs, approximately 230 kDa) and processed gp41 form (gp41-TM11D-scFvs, approximately 110 kDa) were detected in scFv-tethered constructs (Fig. 5A, middle panel). Similar results were obtained with the anti-gp41 Chessie 8 antibody, which can detect both gp160 and gp41 forms (Fig. 5A, lower panel). With Chessie 8, processed gp41from WT and gp41-TM11D-Halo (approximately 80 kDa) of HXB2-TM11D-Halo were also observed. Taken together, these data confirmed the expression and processing of all constructs, although the processing of the Env tethered with foreign protein was not as efficient as for wild type Env.

**Figure 5:** Effect of tethered neutralizing antibodies evaluated by syncytia formation and DSP assay. (A) Immunoblotting analysis of tethered fusion protein expression in 293FT cells with anti-gp120 (upper panel), anti-Flag (middle panel) or Chessie 8 anti-gp41 antibodies (lower panel). The expression vector used is indicated above the lane and the position of different fusion proteins is shown to the right. The anti-gp120 antibody detected the precursor form of tethered proteins and processed gp120 band; the anti-Flag antibody detected the tethered precursor and processed gp41-TM11D-scFv band; and the Chessie 8 anti-gp41antibody detected the processed gp41 (including gp41-TM11D-Halo and gp41-TM11D-scFv) bands. (B) The MFI of different constructs determined by flow cytometry. HaloTag Alexa Fluor 488 ligand was used to stain proteins expressed on the cell surface of 293FT cells transfected with different tethered constructs. The Tac-Halo vector (Halo is expressed in the cytoplasm) was used as a negative control for surface staining. Data was acquired with a BD FACSCalibur system and at least 12,000 events were collected and analyzed using FlowJo software. The MFI of HXB2-TM11D-Halo was set at 100%. Error bars represent standard deviations of the results of triplicate experiments. Student’s *t* test was used for the statistical analysis of the measured variables between individual construct (open column) and control (solid column). Significance was reported with p<0.05(*). ns = nonsignificant. (C) Fusion activity measured by DSP assay. The relative fusion activity was measured by DSP assay. DSP activities for each construct were compared with that of Env tethered with TM11D-MSD and HaloTag (HXB2-TM11D-Halo was set at 100%). Error bars represent standard deviations of the results of triplicate experiments. Student’s *t*-test was used to determine the statistical significance of the measured variables for each construct (open column) and control (solid column). Statistical significance was indicated when p<0.05(*), p<0.001 (***). ns = nonsignificant. (D) Normalization of DSP activity with surface expression level of Env. The DSP activities of each tethered construct shown in panel C were normalized by respective surface expression level defined by MFI measured by flow cytometry shown in panel B. Student’s *t*-test was used to determine the statistical significance of the calculated variables for each construct (open column) and HXB2-TM11D-13H11 (solid grey column). Statistical significance was indicated when p<0.001 (***).

Flow cytometry analysis was performed for cells stained with the HaloTag AF488 ligand to quantify the surface expression level of the tethered fusion proteins. Tac-Halo vector (Halo expressed in the cytoplasm) was used as a negative control [23], [24]. The mean fluorescence intensity (MFI) of different constructs after normalization to that of HXB2-TM11D-Halo is shown in Figure 5B. The attachment of scFv 13H11 showed a higher value of MFI. Although there were some variations among different constructs, the results demonstrated that the MSD of TM11D has a good efficiency to flip out linked foreign proteins.

To examine the effect of the tethered neutralizing antibodies on Env-mediated cell-cell fusion, a DSP assay was performed. As we expected, tethered neutralizing b12 and 2F5 significantly blocked DSP activity compared with Env without scFv (HXB2-TM11D-Halo) or Env with non-neutralizing scFv (HXB2-TM11D-13H11). The raw DSP activity of HXB2-TM11D-13H11 was similar to that of HXB2-TM11D-Halo (Fig. 5C). When we normalized this raw DSP activity with the surface expression level of each tethered Env (Fig. 5D), the significant inhibition of fusion activity was observed for b12 and 2F5. The fusion activity of 13H11 was significantly reduced compared with that of construct without the tethered scFv. This suggests that the addition of scFv itself may have a negative effect on the fusion activity of Env. As shown here, the normalization of the fusion activity with the surface expression level of Env is an important application of our system. Syncytia formation assay also showed tethered b12 and 2F5 totally block syncytia formation, and clear syncytia formation was observed with the tethered non-neutralizing 13H11 construct (data not shown). The expression vector for Env tethered with neutralizing scFv without the second MSD preceding scFv failed to prevent syncytia formation (data not shown). These data suggest that translocated neutralizing scFvs were responsible for the observed blockage of membrane fusion process.

### Critical Residues in scFv for Neutralization can be Mapped using the Tethered Expression System

To further verify the specificity of membrane fusion inhibition by the tethered neutralizing scFvs, we introduced a series of mutations into the tethered scFv domain that suppressed their neutralizing activity. The third complementarity-determining region (CDR) of the heavy chain (H3) of b12 is critical for b12-gp120 binding. Mutations at the tip of this region abolished the binding of b12 Fab with gp120 [37]. We introduced double mutations in this region as depicted in Figure 6A. The DSP analysis indicated a full recovery of the pore formation ability of the mutants, comparable with that of HXB2-TM11D-13H11 (Fig. 6B). The syncytia formation assay also demonstrated the recovery of the cell fusion activity of the mutants, although there was a slight delay in the appearance of syncytia (Fig. 6C). We performed similar experiments using 2F5 constructs. The tip of the CDR H3 loop of 2F5 contains a patch of hydrophobic residues, including residues L100A, F100B, V100D, and I100F (Kabat numbering). A previous study showed that double mutations of these residues to serine abolished 2F5-mediated neutralization (Fig. 6A) [38]. We produced these same double substitutions in our tethered 2F5 construct. DSP assay with these mutants showed no difference with the control HXB2-TM11D-13H11 (Fig. 6B). The syncytia formation assay demonstrated recovery of the ability to form syncytia yet with much slower kinetics: approximately 50% of that of double mutants of L100_A_SF100_B_S, and L100_A_SV100_D_S compared with the control HXB2-TM11D-13H11 at 24 hours after transfection (Fig. 6C). These results suggest that inhibition of syncytia formation with expression vectors bearing b12 or 2F5 is derived from cognitive interactions between scFvs and the corresponding epitopes in Env. Our preliminary results suggested that mutations of the corresponding epitopes in the Env (e.g. mutations in MPER for 2F5) resulted in a similar recovery of syncytia formation (data not shown). Thus, our tethered expression system can be used for the analysis of binding sites in scFv or target Env.

**Figure 6:** Mutations in the CDR3 region of tethered neutralizing scFvs recover fusion activity. (A) B12 and 2F5 CDR H3 loop mutants are listed. Left panel, mutations introduced into the tip of b12 CDR H3 (mutated amino acids are shown in red). The CDR H3 of b12 contains a number of residues important for gp120 binding. These residues are designated D100_A,_ D100_B_. M100_J_ (Kabat numbering). Right panel, mutations introduced in the tip of the 2F5 CDR H3 region (mutated amino acids are shown in blue). The CDR H3 of 2F5 contains a patch of hydrophobic residues affecting its neutralizing activity, including residues L100_A_, F100_B_, V100_D_, and I100_F_ (Kabat numbering). (B) DSP assay with tethered scFv mutants. DSP activities for each mutant scFv construct are shown after normalization to that of the HXB2-TM11D-13H11construct (the activity of 13H11 was set at 100%). Error bars represent standard deviations of the results of triplicate experiments. Student’s *t*-test was used for statistical analysis between each construct (open column) and control (solid column). Statistical significance was indicated when p<0.01 (**). ns = nonsignificant. (C) Syncytia formation assay was performed at the indicated time after the transfection of scFv mutants. The relative fusion activity of mutant constructs was quantified using a fusion index. Fusion activities for each mutant plasmid are shown after normalization to that of the tethered HXB2-TM11D-13H11 expression construct (fusion activity of tethered 13H11 24 h after transfection was set at 100%). Error bars represent standard deviations of the results of observing five fields. Student’s *t*-test was used for statistical analysis between each construct (open column) and control (solid column). Statistical significance was indicated when p<0.05 (*), p<0.01 (**) or p<0.001 (***). ns = nonsignificant.

## Discussion

We tagged HIV-1 Env with HaloTag by introducing an intervening second MSD derived from TM11D. The second MSD relocated the attached HaloTag to the cell surface and allowed the measurement of surface levels of Env by labeling HaloTag with a membrane-impermeable ligand. This modification seemed to reduce the efficiency of processing of gp160 and the surface expression level, but the modified Env still retained fusogenicity. This could be due to the relatively high expression level of Env in our codon-optimized background. Further applicability to the native Env sequences needs to be tested in the future. Non-immunological staining is desirable when diverse field isolates from different clades or laboratory-made mutants that may have different epitopes or structures are dealt with. Our result of the staining with V3-G2-25 illustrates such a possibility. Although raised against NL4-3 that has high sequence homology with HXB2 and JRFL, V3-G2-25 seems to have different efficiency in its recognition of Env of HXB2 and JRFL. This study demonstrated live cells could be labeled with HaloTag ligand with high efficiency using a simple procedure. Furthermore, HaloTag ligand-labeled Env retains fusogenicity. Therefore the labeled Env can be directly applied to the fusion assay. This retention of fusogenicity after labeling cannot always be expected when using immunological staining.

To our knowledge, this is the first report using the MSD of TM11D, a type II membrane protein, to connect two different proteins in tandem and alter the membrane topology of the connected protein. In addition to the MSD of TM11D, we also tested a simple hydrophobic sequence or other MSD derived from type I and II membrane protein. Our preliminary data suggested that the MSD of TM11D was better than other tested sequences. However, whether the MSD of TM11D would work well in other contexts needs to be evaluated further.

Our data showed that the additional peptide or protein sequence could be linked after the C-terminus of HaloTag. By adding C34 or neutralizing scFvs, we observed the inhibition of membrane fusion. It is noteworthy that stoichiometry between the attached peptide/protein and Env was fixed to 1∶1 in our system. Studies involving the co-transfection of two expression vectors or addition of the exogenous peptides may not be able to achieve this kind of fixed stoichiometry. Furthermore, since the synthesis of oligonucleotides is more cost effective than that of peptides, our system may provide an alternative method to evaluate many candidate fusion inhibitory peptides. Other researchers have analyzed C-peptides including C43, C34, and C28; consistent with our results, the shortest active peptide was C28 [26], [39], [40], [41]. Furthermore, our results clearly showed the length of C-peptide correlated well with the fusion inhibitory effect: C24 showed 30% recovery of the membrane fusion ability compared with HXB2-TM11D-Halo construct (Fig. 4A, 4B).

We also tethered scFvs in our system and showed that characterization of scFv could be achieved as for the inhibitory peptides. This method allows the adjustment of the fusion ability of Env by its surface expression level (Fig. 5D). This adjustment with the surface level of Env may be more useful than normalization with the total Env level revealed by immunobloting analysis. Using our tethered expression system, we can bypass the steps of expression and purification of scFv, which are often a major time-consuming factors in the scFv system [42], [43], [44], [45]. Preliminary analysis indicated that epitope mapping of the target Env was also possible (data not shown).

Interestingly, although pore formation detected by DSP assay was recovered for both b12- and 2F5-scFv mutants to a similar level to the wild type, there was a difference in the ability to recover syncytia formation in two scFvs (Fig. 5A, 5B). The 2F5-scFv mutants showed poor recovery of syncytia formation even after 24 hours post transfection. The mechanism of inhibition of HIV-1 infection by 2F5 antibody has not been completely elucidated. A previous study demonstrated that 2F5 mutants (also used in this study) changed the hydrophobicity of the apex loop of 2F5, while another study argued the L100_A_AF100_B_A mutant (the same position as our mutation) leads to a reduction in binding to lipid vesicles [38], [46], [47], [48]. Our data suggest that some steps after pore formation, such as pore dilatation, could be affected by interactions between Env and 2F5-scFv.

Several previous reports showed that the weak or non-neutralizing antibodies were converted into broadly neutralizing antibodies when scFv and Env were co-localized intracellularly [49], [50], [51], [52], [53]. In our system, Env and a candidate scFv co-localized with fixed stoichiometry and may interact intracellularly. Therefore it is possible that our tethered system may provide a unique microenvironment to identify some scFvs with weak fusion inhibitory activity.

In this study, we generated an expression system that allowed the simultaneous expression of HIV-1 Env and foreign peptides or proteins on the cell surface by connecting them to an intervening MSD. Although it is a very artificial expression system, it may provide a useful tool to study membrane fusion mechanisms. Membrane proteins other than HIV-1 may be adopted into this tethered expression system to facilitate their characterization.

## Materials and Methods

### Plasmid Construction

HXB2-TM11D-Halo was modified from pHIVEnv which expresses codon-optimized HXB2 Env (HXB2-WT) by adding MSD of TM11D and HaloTag to downstream of env [23], [24]. A polynucleotide containing multiple cloning sites and fragments corresponding to amino acid polylinkers was synthesized (Taihe Biotechnology, Beijing, China) and cloned into pHIVEnv using *Sal*I and *Xba*I sites. A polynucleotide corresponding to MSD of human transmembrane protease serine 11D (TM11D MSD) was synthesized (Taihe Biotechnology) and cloned into pHIVEnv via *Not*I and *Xba*I sites. The amino acid sequence of TM11D MSD is FIVVAGVVILAVTIALLVYFI. HaloTag was extracted from plasmid pFC15A-HaloTag7-CMVd1 (Promega, WI, USA) by PCR, and was cloned into pHIVEnv via *Xho*I and *Acc65*I sites. Codon-optimized JRFL *env* was synthesized (Taihe Biotechnology, Beijing, China) and cloned into pHIVEnv and HXB2-TM11D-Halo via *Eco*RI and *Sal*I sites to generate JRFL-WT and JRFL-TM11D-Halo, respectively.

To generate the HXB2-TM11D-C34 construct, the C34 gene was synthesized and cloned into a pGSI vector at *Bsi*WI and *Kpn*I restriction enzymes sites (Taihe Biotechnology). Then the C34 gene was cut out with *Bsi*WI and *Kpn*I restriction enzymes and inserted into the 3′ of a HaloTag sequence in the HXB2-TM11D-Halo vector.

C34 serially truncated mutants were generated using a QuikChange Site-Directed Mutagenesis kit (Stratagene, La Jolla, CA, USA). The C34 sequences cloned into the pGSI vector were used as a template for mutagenesis. The generated truncations were cloned into a pHXB2-TM11D-Halo plasmid using *Bsi*WI and *Kpn*I sites.

To generate tethered antibody display constructs, genes corresponding to the heavy and light chains of scFv fragments of monoclonal antibodies b12, 2F5 and 13H11 were synthesized (Taihe Biotechnology) and cloned to the corresponding positions of a pIT2 phagemid vector. pIT2 phagemid vectors were obtained from Human Single Fold scFv Libraries I+J (Tomlinson I+J) (Source BioScience, LifeSciences, UK). To generate the tethered scFv expression construct, genes encoding b12, 2F5, and 13H11scFvs in the pIT2 phagemid vector were amplified by PCR using the forward primer BsiF (5′-CGTACGGCCCAGCCGGCCATGGCC-3′) and different reverse primers: b12KpnR (5′-GGTACCTGCGGCCGCAGTACGTTTA-3′), F5KpnR (5′-GGTACCTGCGGCCGCAACAGTACGA-3′), 13H11KpnR (5′-GGTACCTGCGGCCGCCACGGTGCG-3′). PCR products were cloned into a pGEM-T vector (Promega). After sequence verification, the scFv genes were cut out with *Bsi*WI and *Kpn*I restriction enzymes and inserted to the 3′ of a HaloTag sequence in the HXB2-TM11D-Halo vector. The DNA sequence of 3×FLAG was synthesized (Taihe Biotechnology) and connected to the 3′ end of the scFv gene in the tethered construct.

ScFv mutants’ constructs were produced using a QuikChange Site-Directed Mutagenesis kit (Stratagene). The scFv sequences cloned into the pGEM-T vector were used as a template for mutagenesis. The generated mutant scFvs were cloned into the HXB2-TM11D-Halo plasmid using *Bsi*WI and *Kpn*I sites.

### Generation of Stable Cell Lines Expressing Individual DSP

To establish stable cell lines expressing DSP_1–7_ and DSP_8–11_, each DSP gene prepared by PCR was cloned into a mammalian expression vector, pIRESpuro3 (Clontech). The DSP genes were prepared by PCR as follows. DSP_1–7_ ORF was amplified by PCR from pCMV-DSP_1–7_, 5′-AGAGCGCTAGCATGGCTTCCAAGGTGTACGACC-3′, and 5′-GATGCGGATCC TTACTTGTCGGCGGTGATGTAC-3′ as the forward and the reverse primers. DSP_8–11_ ORF was amplified by PCR from pCMV-DSP_8–11_, 5′-AGAGCGCTAGCATGCAGAAGAACGGCATCAAG-3′ and 5′-GATGTCCCGGGTTACTGCTCGTTCTTCAGCAC-3′ as the forward and the reverse primer, respectively.

Transfection of pIRESpuro3-DSP_1–7_ and pIRESpuro3-DSP_8–11_was performed with 293FT and 293 CD4 cells using the Neon transfection system (Invitrogen, Carlsbad, CA, USA). After 48 h incubation in Dulbecco’s modified Eagle’s medium (DMEM) (Sigma, St. Louis, MO, USA) supplemented with 10% fetal bovine serum (FBS; Thermo Scientific HyClone, UT, USA), 1.5 µg/ml of puromycin was added to the culture and selection was performed for 10–13 days.

### Cell Culture and Transfection

293FT cells (Invitrogen) or 293CD4 cells (293 cells constitutively expressing human CD4) [30] were grown in DMEM supplemented with 10% FBS. Cells were kept under 5% CO_2_ in a humidified incubator (Sanyo, Japan) and then transfered to a 6- or 96-well-plate (BD Falcon, San Jose, CA, USA) 1 day before transfection and Fugene HD (Promega) was used for transient transfection.

### Immunoblotting

293FT cells (2×10^5^) were transiently transfected with pHIV Env and tethered expression vectors by FuGENE HD in a 6-well culture plate. Cells were lysed with 60 µl RIPA lysis buffer (Thermofisher Scientific, MA, USA) at 48 h after transfection. After centrifugation at 20,400×*g* for 30 min at 4°C, the supernatant was collected and the protein concentration was determined by Pierce BCA protein assay (Pierce Biotechnology, Rockford, USA). Samples containing about 50 µg proteins were loaded into each well, electrophoresed (10% SDS-PAGE, Bio-Rad Ready Gel J) and transferred to a polyvinylidene fluoride membrane (Millipore, Immobilon-PSQ). The blot was probed with anti-gp120 polyclonal antibody (Fitzgerald, Concord, MA, USA), monoclonal anti-FLAG antibody (Sigma-Aldrich), or monoclonal antibody Chessie 8 [54]. Donkey anti-Goat IgG-HRP (Santa Cruz Biotechnology, Santa Cruz, USA) or goat anti-Mouse IgG-HRP (Santa Cruz Biotechnology) was used as secondary antibodies. The blot was further treated with ECL Western Blot Kit (CWBIO, Beijing, China). Images were obtained with LAS3000 (Fujifilm, Tokyo, Japan).

### Labeling HaloTag with Specific Ligands

At 48 h after transfection, HaloTag ligands were added to the transfected 293FT cells according to the manufacturer’s instructions. Briefly, transfected cells were labeled for 15 min at 37°C with 1 µM of HaloTag ligand TMR, Alexa Fluor 488 (AF488) or Oregon Green. After labeling, cells were rinsed three times with 200 µl prewarmed DMEM/FBS and subsequently incubated at 37°C under 5% CO_2_ for 30 min. After the medium was replaced with fresh warm DMEM/FBS, images were captured using a confocal microscope (Olympus FV1000, Tokyo, Japan).

### Flow Cytometry

293FT cells (1×10^5^) were transfected with the construct of interest in triplicate. At 48 h post-transfection, HaloTag Alexa Fluor 488 Ligand (Promega) was used to label HaloTag as described above. After washing with phosphate-buffered saline (PBS), cells were detached and resuspended in PBS with 3 mM EDTA, followed by 4% paraformaldehyde fixation; alternatively, 1 µg/mL V3-G2-25 antibody [25] was added to the cells after PBS washing and incubated at 4°C for 30 min. Then washed cells were incubated at 4°C for 30 min with 1 µg/mL Alexa Fluor 488 donkey anti-mouse IgG antibody (Invitrogen). Finally, the cells were resuspended in PBS with 5% FBS and 4% paraformaldehyde. Flow cytometry data were acquired with a BD FACSCalibur system (Becton, Dickinson and Company), at least 10,000 events were collected and analyzed using FlowJo software (Tree Star).

### Fusion Assay (Syncytia Formation Assay)

Fusion activity was evaluated by syncytia formation assay. Expression vectors were transfected into 293CD4 cells by FuGENE HD (using a 5∶2 ratio of FuGENE HD transfection reagent to DNA [µl/µg]), and visible syncytia formation was evaluated at 16–24 h post-transfection. To visualize syncytia formation, Hoechst 33342 and CellMask Deep Red plasma membrane stain (Invitrogen) were used to stain nuclei or membranes, respectively. The transfected cells were labeled for 15 min at 37°C with CellMask Deep Red plasma membrane stain (5 µg/ml) and Hoechst (0.2 µg/ml). After labeling, the cells were rinsed three times with 200 µl pre-warmed DMEM/FBS and images were captured using a confocal microscope (Olympus FluoView FV1000). The fusion index was calculated to estimate the degree of syncytia formation. The fusion index = 2x+y was calculated by examining five random fields under a microscope, where x is the number of multinucleated cells [number of nuclei ≥5], and y is the number of multinucleated cells [number of nuclei <5].

### Fusion Assay using Dual Split Protein (DSP)

For the fusion assay, cell lines stably expressing DSP were utilized (see above), the stable cell line expressing dual split protein DSP_8–11_, were transfected with expression vectors of interest in quadruplicate. At 48 h post-transfection, 293CD4/DSP_1–7_ cells (2×10^4^), a stable cell line expressing CD4 and DSP_1–7_, were co-cultured with transfected 293FT/DSP_8–11_ cells at 37°C in fresh medium containing membrane-permeable Enduren Live Cell Substrate (Promega). The RL activity was measured at 2hr after co-culture using GloMax-Multi Plus Detection System (Promega).

For designated experiments, the same batch of transfected 293FT/DSP8-11 cells were subjected to FACS analysis as described above. The RL activity readings were normalized to the respective MFI to compensate for the differential surface expression level of Env.

For DSP assay of cells after staining with Halo ligand, transfected cells were labeled for 15 min at 37°C with 1 µM of HaloTag TMR or Alexa Fluor 488 ligand. After labeling, cells were rinsed three times with 200 µl prewarmed DMEM/FBS and subsequently incubated at 37°C with 5% CO_2_ for 30 min. After the medium was replaced with fresh warm DMEM/FBS, images were captured using a microscope, then this sample was used directly for DSP assay.
